# Research Progress on Therapeutic Effect and Mechanism of Propolis on Wound Healing

**DOI:** 10.1155/2022/5798941

**Published:** 2022-07-21

**Authors:** Juan Yang, Anjuan Pi, Lele Yan, Juan Li, Sha Nan, Jing Zhang, Yuhui Hao

**Affiliations:** ^1^Department of Biochemistry and Molecular Biology, Chongqing Normal University, College of Life Sciences, Chongqing 400000, China; ^2^State Key Laboratory of Trauma, Burns and Combined Injury, Institute of Combined Injury, Chongqing Engineering Research Center for Nanomedicine, College of Preventive Medicine, Army Medical University, Chongqing 400000, China

## Abstract

Propolis is a kind of reduct collected by bees from various plant sources. Because propolis is a mixture, it has a variety of biological activities, excellent anti-inflammatory and bactericidal effects. Especially in the treatment of infectious wounds, acute wounds, burns, and scalds and promoting wound healing, more and more scientists began to apply it to the research field of wound healing. The standard preparation of propolis combined with other compound components has a safer and less toxic effect in the treatment of trauma. In order to more effectively use propolis products in wound treatment. This paper reviews the effect and treatment mechanism of propolis on different types of wound healing, as well as the synergistic effect of propolis and other compounds, in order to provide ideas for the further exploration of the biological activity and pharmacological function of propolis in the future, as well as its in-depth development in the field of wound healing. It will also provide a theoretical reference for the further development and utilization of propolis.

## 1. Introduction

In a broad sense, trauma refers to body injuries caused by physical, chemical, and biological factors, including knife injuries, crush injuries, and frostbite. Trauma has a high incidence in the population. People have done a lot of research on drugs for wound repair from the perspectives of anti-inflammatory, antibacterial, antioxidant, and antiseptic [1]. Many drugs for treating local trauma have been developed, but most drugs have single pharmacological activity and may have certain side effects on the body [2, 3]. Silver sulfadiazine (AgSD), a silver compound, is often used to prevent or treat wound colonization, and also certain antibiotic-resistant bacteria. In vitro studies have shown that when acute rat wounds are used as a model, the topical antibacterial agents silver sulfadiazine and mafenyl acetate can destroy fibroblasts and have toxicity. This indicates that silver sulfadiazine and mafenyl acetate can significantly hinder wound contraction in the body [4–6]. Some researchers have found that when sulfadiazine is used to treat burns in experimental mice, it will also produce greater inflammatory reactions, such as redness and swelling [7]. Vaseline was used as the control group to treat the wounds of mice. Compared with the drug treatment in the experimental group, the wounds healed more slowly [8]. In a large number of studies, propolis, as a natural product that can promote tissue healing, has various biological activities, such as anti-inflammatory, antibacterial, and antioxidant. It has obvious advantages in promoting wound repair and has achieved ideal therapeutic effects. This kind of wound healing refers to the healing process after the body is broken or damaged by external forces, skin and other tissues, including the regeneration of various tissues and the complex combination of granulation tissue hyperplasia and scar formation, showing the synergy of various repair processes.

Propolis has always been considered as a folk medicine. Its research can be traced back to ancient times, and it was discovered about 300 years ago. Propolis is usually a sticky substance, which is formed by the resin collected from trees by Italian worker bees and the secretion of their maxillary glands. Propolis is extremely complex and contains a variety of compounds, such as flavonoids, terpenes, phenolic acids, aldehydes, and ketones, as well as a variety of hydrocarbons, minerals, trace elements, vitamins, and enzymes. Twelve different flavonoids, namely, pinocembrin, acacetin, chrysin, rutin, luteolin, kaempferol, apigenin, myricetin, catechin, naringenin, galangin, and quercetin; two phenolic acids, caffeic acid and cinnamic acid [9] (Figure 1). Propolis is a kind of mixture, which contains a variety of chemical components, but its most active chemical substances can also play a role alone. Phenethyl caffeic acid extracted from bee propolis is a receptor activator that regulates oxidation state and NF-kB ligand (RANKL)/osteoprotegerin (OPG) signal, and has potential protective effect on glucocorticoid induced osteoporosis (GIO) [10]. It can also promote collagen deposition, re-epithelialization and wound healing in mice 12 days after pressure ulcer. In addition, it also promoted the inflammatory response, oxidative stress, and NRF2 expression, and made the skin wound of pressure ulcer in mice heal [11]. In order to determine the relationship between polyphenol derivatives in propolis and their antioxidant and antibacterial activities, some researchers studied the propolis extract from Bihor County, Romania. Different ethanol concentrations were used to extract propolis. The total polyphenols measured ranged from 1.5 to 91.2 mg/g. The final results showed that 50% ethanol extract provided rich polyphenols and ensured good antioxidant capacity [12]. In addition to caffeic acid phenethyl ester and polyphenols, there is also an important single-substance flavonoids. chrysin (CR) is a flavone, which exists in propolis and many plants. Populin was used to treat LPS-induced sepsis in rats, which could reduce the levels of oxidative stress markers and cytokines in patients with sepsis [13]. With the deepening research on propolis by scholars at home and abroad, the biological and pharmacological activities of propolis have been further revealed. It plays an important role in antioxidation, scavenging free radicals, antibacterial and anti-inflammatory, protecting the liver, improving human immunity, antitumor, oral health, regulating blood lipids, gastrointestinal diseases, anti-vascular effects, reducing blood glucose, and so on [14] (Table 1).

Studies have shown that different forms of propolis have an effect on wound healing (Table 2). According to these results, it can be seen that propolis has a significant effect on various wound treatments. On the basis of previous studies, this paper summarizes the effect and related mechanism of propolis on wound healing and the synergistic effect of propolis and other compounds, which further clarified the medicinal value of propolis and provided a more powerful basis for propolis theory.

## 2. Effect of Propolis on Wound Healing

The skin is the largest organ of the human body. When it comes into direct contact with the external environment, it is often damaged by a variety of physical, chemical, and biological factors. Minor trauma is limited to skin surface injury, while severe trauma may include rupture and fracture of muscles, tendons, and nerves. As the body's first-line of immune defense, it is easily invaded by bacteria after being destroyed, causing wound infections. Therefore, the skin should be treated promptly after trauma. Classical wound healing is divided into inflammatory stage, tissue growth stage, and tissue remodeling stage [46]. The repair method and time are determined by the degree of injury, the ability of tissue regeneration, whether the wound has necrotic tissue and foreign bodies, whether there is infection and other factors. Propolis has a unique effect on the healing of trauma and surgical knife edge. It has many effects, such as pain relief, antibacterial, promoting skin regeneration on the wound, promoting granulation growth, limiting scar formation, and so on. It is much superior to the methods in other stages currently used.

### 2.1. Effect of Propolis on Acute Trauma

Acute trauma is a trauma caused by a direct or indirect external force. It is generally caused by trauma, war injuries, and emergencies, including burns, lacerations, abrasions, and surgical wounds. With the rapid development of industry, agriculture, transportation, and sports, the trauma caused by various accidents is increasing. Trauma not only has a high incidence, but also varies greatly in degree. The injury can be serious and complicated, and even endanger the life of the wounded. Severe trauma can cause systemic reactions, local manifestations include pain, swelling, tenderness in the injured area, deformity, and dysfunction in case of fracture and dislocation. Severe trauma may also have fatal bleeding, shock, asphyxia, and disturbance of consciousness. Therefore, it is necessary to use the physiological activity characteristics of propolis to treat acute wounds.

#### 2.1.1. Burn

Generally, burn wounds have to go through three stages: inflammation, tissue hyperplasia, and scar formation. The early inflammatory response largely determines the development of later scars. For the human body, the largest organ is the skin, and the normally healed wound after trauma will not affect the function. Only in case of severe trauma or abnormal inflammatory response, the tissue is over repaired, resulting in scar tissue, affecting the beauty and even causing canceration [47, 48]. Some researchers used pigs as experimental subjects and caused 72 contact burns on the left and right sides of pigs. In the process of collagen extraction, propolis ointment can stimulate the extraction rate of collagen more than other preparations. The expression of collagen and its components was significantly increased. In addition, the increased accumulation of collagen in the damaged matrix cured with propolis may stimulate the repair process [3]. Burned rats were treated with 5% propolis every day, which cured second degree burns in the neck area of female rats due to metal scald. Propolis treatment accelerates the process of tissue repair and leads to the reduction of local inflammation, which indicates that propolis treatment is successful. The production of collagen fibers was stimulated at all evaluation stages by morphometry. The authors believe that propolis treatment can restore function faster and finally improve the quality of life of burn patients [49]. Some researchers have also explored the applicability of collagen membrane of water alcohol extract of red propolis and green propolis to skin burn healing in rodent model. The water and alcohol extracts of the two were combined with collagen-based dressing membrane for burn wounds on the back of rats. The inflammatory response, epithelial formation rate, myofibroblast count, and collagen formation were evaluated histologically at several time points during wound healing. The results showed that the water and alcohol extracts of the two propolis could reduce the degree of inflammation. In addition, propolis showed no toxicity during treatment, indicating that propolis had a good effect on wound healing [50]. Some people have studied the dynamic changes of vitronectin, laminin, and heparan sulfate/heparin during the healing process of experimental burns. The wounds were treated with propolis, silver sulfadiazine (AgSD), normal saline, and propolis carrier. After burns, the content of adhesion protein increased, and after treatment with propolis, it showed a significant decrease. Compared with several other preparations, propolis can stimulate wound healing faster and reduce inflammation. This also reveals the potential role of propolis in promoting wound healing [51].

#### 2.1.2. Other Acute Wounds

Common acute wounds can also appear at any time in life, such as lacerations, abrasions, and postoperative wounds. For some small wounds, the repair ability of the body tissue can heal itself, but for serious and complex wounds, medication must be used. Some researchers used a combination of technology to encapsulate propolis in a self-microemulsification formula to treat trauma in rats. Release studies have shown that propolis markers can be released continuously for up to 7 days. This new type of dressing is based on a self-microemulsified drug delivery system that co-encapsulates propolis and cinnamon essential oil in BC to achieve a polysaccharide film with high antimicrobial activity to promote wound healing [43]. In this study, four kinds of propolis-containing extracts and one kind of nano-metal particles without propolis were prepared by microwave method, and their wound healing activity in the experimental model of rat wound resection was evaluated. It proves the possibility of this new material dressing containing propolis for wound care. Compared with other nanoparticles, it has a significant effect [52]. Someone also studied silk threads coated with propolis and bio-silver nanoparticles, and conducted characterization studies. This antibacterial suture material with enhanced wound healing function can protect the surgical site from infection [31]. Nigerian propolis was used as a wound healing agent to treat full-thickness skin wounds in healthy adult male albino rats. According to the wound healing index, Nigerian propolis extract can accelerate wound healing, similar to silver sulfadiazine (AgSD), which can be used for medical treatment [53]. In addition, an external preparation (apavash ointment) containing Brazilian micro-propolis extract and Peucedanum leaf extract was used to treat the wounds caused by surgical perforation in rats. After two weeks of experiment, the experiment was divided into four groups: gauze group, polyethylene glycol basic ointment group, apavash ointment group, and polysporomycin group. The final result was that the apavash ointment group and the polysporomycin group showed some additional benefits, using myeloperoxidase and histological counts, as well as fibrosis and hydroxyproline production. The results showed that both of the two treatments could promote wound healing and form better skin quality [54].

The resected wounds of experimental rats were treated with Indian propolis ointment to evaluate its healing potential. Compared with the control group, the wound contraction was significantly improved. The levels of hydroxyproline, hexosamine, uronic acid, DNA, RNA, and protein in wound matrix increased significantly. Therefore, the authors concluded that the ethanol extract of Indian propolis has significant healing promoting activity by accelerating the healing process at different stages of tissue repair [8]. In addition, two square skin incisions were made in the neck of the rats and treated daily with a preparation containing propolis ointment. Compared with the control group, the propolis ointment affected the healing process of stimulating the proliferation of keratinocytes. It shows the promoting effect of propolis ointment on wound healing [30]. In addition, the effects of oral propolis alone or combined with nano-silver on wound healing in male rats were also studied. The control group was not treated, and the experimental group was divided into three groups. Propolis alone and propolis combined with two different concentrations of nano silver ions were taken orally. The healing rate was determined by the reduction of wound surface area on postoperative days 4, 6, 8, and 10. The results showed that the wound healing of the control group and the experimental group was significantly different, especially, the fibroblast count of propolis + 30 ppm SNPs group was the highest, and the difference of collagen fiber density was also significant. Finally, the authors concluded that oral propolis alone in combination with 30 ppm SNPs can provide anti-inflammatory effects and increase fibroblast proliferation and collagen deposition in experimental wounds, which may explain the observed healing differences [55].

### 2.2. Effect of Propolis on Chronic Trauma

Chronic trauma generally refers to the trauma accumulated by small trauma due to repeated attacks caused by improper treatment after acute injury, or constant strain during exercise. The symptoms of chronic wounds are slow, the course of disease is prolonged, and skin and soft tissue defects cannot be repaired in time. It includes oral ulcer, diabetic foot ulcers, and venous ulcers of the lower extremities. Propolis also plays an important role in the treatment of chronic wounds.

#### 2.2.1. Oral Ulcers

Oral ulcers are a common oral mucosal problem. The patient suffers severe pain during the onset. In severe cases, it affects eating and speaking, causing great inconvenience to life. What effect does propolis have on oral ulcers? In a diabetic rat model, Indonesian scientists concluded that the application of propolis extract gel to oral mucosal traumatic ulcers can reduce the expression of MMP-9, increase the expression of vascular endothelial growth factor (VEGF), and accelerate the healing process [56]. In the experiment of using propolis to study oral ulcers, propolis was not only applied to animals, but also was used to treat human oral ulcers. Israeli researchers have launched a clinical trial using propolis to apply propolis to the affected area of a girl with a serious oral ulcer problem and ineffective long-term treatment. The test found that after applying propolis for 10 days, the area of the ulcer was significantly smaller and narrower. After applying propolis for 3 weeks, the oral ulcer was completely healed, and the oral ulcer did not recur in her subsequent life [57]. Recurrent aphthous stomatitis is also a common, painful, ulcerative oral disease. Patients take 500 mg of propolis a day. After six months of experimentation, the quality of life of patients taking propolis has improved significantly. The final results show that propolis can effectively reduce the recurrence of recurrent oral ulcers and improve the quality of life of the patients [58]. The Brazilian green gum gel is used to treat patients with denture stomatitis, and the drug is continuously administered four times a day for one week. Brazilian propolis gel has mucosal adhesion properties and can promote the healing of the affected parts of all patients. None of the patients showed any signs or symptoms of allergies or allergies [59]. 

#### 2.2.2. Venous Leg Ulcers

Chronic venous ulcers of the lower extremities are serious and intractable manifestations of chronic venous insufficiency of the lower extremities, and the prevalence in the population is as high as 1.1–1.8%. There are many factors that cause venous ulcers. It is believed that the most important pathogenesis is venous hypertension caused by abnormal venous blood flow. The pathophysiological basis of venous ulcers is venous hypertension of the lower extremities. Either venous return obstruction or venous backflow can lead to venous hypertension. Venous ulcer of lower limbs, commonly known as “old rotten leg”, is mainly a chronic skin ulcer in the middle and lower leg. Some researchers used propolis ointment to locally administer lower extremity venous ulcer, and evaluated its curative effect. Fifty-six patients were divided into two groups. One group was treated with topical propolis ointment application and short stretch bandage compression, and the other group was treated with Unna's boot leg compression surgery without topical propolis treatment. The two groups healed completely in the sixth week and the sixteenth week, respectively. It is obvious that the use of propolis to treat wound healing time significantly speeds up, an auxiliary propolis ointment treatment increases the efficacy of short stretch bandage compression stockings, this combination treatment is more effective than using Unna's boot compression stockings alone [60].

#### 2.2.3. Diabetic Foot Ulcer

Diabetic foot ulcer is an ischemic, neurological, and neuroischemic pathology of the foot caused by diabetes. It can cause different degrees of infection, ulcers, and gangrene in the foot, and increase the risk of amputation. It is one of the common complications of diabetes. In diabetic patients, there is a 15–20% chance of suffering from diabetic foot [61]. Some researchers have studied topical propolis to promote wound healing in patients with diabetic foot ulcers. Finally, within 4 weeks after topical application of 5% propolis ointment, the area of the ulcer was reduced and the wound healing process was enhanced [31]. There are also patients who used propolis to treat diabetic foot ulcers. The propolis group and the treatment group were completely healed in the third and seventh weeks, respectively, and the active MMP-9 of the propolis group was significantly reduced after debridement [62]. Another research team revealed the molecular mechanism of improved diabetic wound healing after propolis treatment. The results showed that after treating the wound with propolis, it significantly promoted the healing of the wound in diabetic mice. Propolis promotes tumor growth factor *β* (TGF-*β*) signal transduction, significantly reduces the levels of matrix metalloproteinases and pro-inflammatory cytokines in the wounds of diabetic mice, and enhances the deposition of type I collagen [63]. In addition, some researchers have evaluated the role of propolis as an adjuvant in the healing of human diabetic foot ulcers. Dynamic healing of diabetic foot wounds with propolis spray. At the same time, the macroscopic and microscopic aspects of the wound healing process were analyzed. Compared with the control group, propolis promoted an average reduction of 4 cm^2^ in wound area, which was related to the increase in connective tissue deposition. In addition, propolis increased the ratio of glutathione and glutathione/glutathione disulfide, and decreased TNF-*α* and increased IL-10 [64].

## 3. The Possible Mechanism of Propolis on Wound Healing

The mechanism of wound healing by propolis mainly includes the following five aspects: antibacterial, anti-inflammatory, antioxidant, immune, and mast cell (Figure 2).

### 3.1. Anti-inflammatory Effect

Inflammation is a kind of defense response of the body to stimulation, which is characterized by redness, heat, pain, and dysfunction. It can be infectious inflammation caused by infection or non-infectious inflammation caused by infection. After experiencing burns and trauma, severe symptoms are manifested by a large number of degenerated and necrotic tissues, bacterial invasion, massive production of free radicals, and inflammation caused by stress response [65]. Scientists have found that propolis can alleviate inflammatory problems and promote wound healing. The anti-inflammatory biological activity of propolis is mainly related to the fact that propolis contains a large number of flavonoid anti-inflammatory substances, such as carnitine and galangin, as well as phenolic anti-inflammatory substances, such as caffeic acid, ferulic acid, phenethyl caffeic acid, and so on [66]. A large number of in vivo experiments on the repair activity of propolis have observed that propolis promotes wound repair, accompanied by inhibition of local inflammatory response of wound (Table 3).

Some researchers knocked out the smad3 gene in mice, which abnormally showed accelerated skin wound healing compared with wild-type mice. The results showed that the local mononuclear cell infiltration of the mouse wound was significantly reduced, and the re-epithelialization speed increased, reflecting the inhibitory effect of the inflammatory response on the re-epithelialization [71]. Dietary propolis has an effect on the metabolism of arachidonic acid in vitro and in vivo. It significantly inhibits the lipoxygenase pathway of arachidonic acid metabolism in the process of inflammation in the body [72]. Propolis ethanol extract may exert its anti-inflammatory effect by inhibiting the expression of iNOS gene, by acting on the iNOS promoter at the NF-kB site and directly inhibiting the catalytic activity of iNOS [73]. There is another possibility that the anti-inflammatory effect of propolis may be caused by the carbon monoxide mechanism [74].

In general, inflammatory response can play a positive role in wound repair through anti-infection, tissue debridement and release some cytokines, but it will also inhibit some aspects of tissue repair.

### 3.2. Antibacterial Effect

Bacterial infection is an acute systemic infection caused by pathogenic bacteria or conditional pathogenic bacteria invading the blood circulation, growing and reproducing, producing toxins and other metabolites. Clinically, it is characterized by shivering, high fever, rash, joint pain, and hepatosplenomegaly, some patients may have septic shock and transitional lesions.

Since ancient times, humans have used the antibacterial properties of propolis, including as a wound healing promoter [75]. A large number of experiments have also shown the antibacterial properties of propolis (Table 4). At present, the research on the mechanism of antibacterial activity is not clear, and it may be combined with some other biological materials to play a role. Some researchers also pointed out the antibacterial activity of propolis ingredients, polyphenols and flavonoids against *Escherichia coli* and *Staphylococcus aureus* [80]. Studies have also shown that propolis extract drug-loaded preparations can inhibit *Staphylococcus aureus* and *Staphylococcus epidermidis* [38]. In addition, propolis also has a good antibacterial effect on negative bacteria such as *Escherichia coli* and *Pseudomonas aeruginosa* [81]. The amino acids, vitamins, and carbohydrates contained in propolis, can provide local nutrition for wounded tissues and improve the microenvironment of local tissues [82]. This may be one of the reasons why it promotes tissue repair. Propolis has a good antibacterial activity, no side effects of general antibiotics, and does not produce drug resistance. The effect of propolis on Gram-positive bacteria is stronger than that on Gram-negative bacteria, especially for *Staphylococcus aureus*. Some researchers have studied the characteristics of silk thread coated with propolis and biological silver nanoparticles, which is based on the wound healing of surgical site infection. Bioactive propolis coated suture showed effective antibacterial activity against pathogenic Gram-negative and Gram-positive bacteria, *Escherichia coli* and *Staphylococcus aureus* [45].

### 3.3. Antioxidation Effect

Oxygen is an indispensable element for human life activities. However, while oxygen reacts in the human body to provide heat energy for the human body, some oxygen will produce hydrogen peroxide, superoxide anion, and free radical hydroxyl. These excess free radicals will act on the cell membrane and lipid substances in blood to form lipid peroxides. They will deposit on the cell membrane, resulting in the loss of membrane function and the decline of cell vitality, resulting in human aging. Propolis is recognized as a natural antioxidant because it is rich in flavonoids, unsaturated fatty acids, VE, VC, and trace elements such as zinc and selenium.

After severe burns, mediators including reactive oxygen and reactive nitrogen increase in the affected tissues [83]. The rich flavonoids, phenolic acids, and mushroom alkenes in propolis make it have a good antioxidant effect. Therefore, this is probably one of the important reasons for propolis to promote wound healing. There are also experiments to prove the antioxidant activity of propolis (Table 5). These antioxidant active substances can directly scavenge free radicals or increase the activity of some antioxidant enzymes in the cell, and even exert their antioxidant activity by affecting the signal transduction process of oxidative-stress-related transcriptional regulators [87]. Researchers studied the effects of propolis on free radicals in burn tissues and detected the concentration of free radicals in burn tissues in the propolis treatment group by electron paramagnetic resonance spectroscopy. The results showed that propolis can make the concentration of free radicals in burn tissues relatively low [88]. Some researchers made propolis into local liposomes for wound treatment and tested its antioxidant capacity. The results showed that the antioxidant activity was not related to the concentration of propolis in ethanol solution, which may be the result of the stability of antioxidants and even oxidants in propolis. In addition, F3 liposome formulation showed higher antioxidant activity than S3 solution. The results showed that the empty liposome preparation may also have significant antioxidant activity [89]. The antioxidant activity of some propolis samples collected from Palestine and Morocco was determined. The measured propolis samples showed stronger DPPH radical scavenging activity, with EC50 between 0.14 ± 0.01and 0.02 ± 0.01 mg/ml. Moreover, the content of total phenols and flavonoids/flavonols in the sample was high, so it has strong antioxidant and antibacterial properties [90]. When Tigzirt propolis was tested for anti-inflammatory and antioxidant effects, it was found that propolis extract helped to reduce PGE2 and TNF-*α*、Myeloperoxidase and malondialdehyde levels, and increase the total antioxidant level in plasma [91].

These studies suggest that propolis and its active components may increase or restore the activity of some antioxidant enzymes in traumatic tissue, and promote the increase of its content and the direct scavenging effect on free radicals, protect cells from oxidative damage, so as to promote tissue repair. In addition, some researchers have found that H_2_O_2_ released outside the cell can pass through the plasma membrane through specific aquaporins (AQP3) that regulate intracellular reactions. AQP3-promoted water transport plays a key role in cell migration and accelerates skin wound healing. Their results showed that reactive oxygen species (ROS) produced by propolis exposure could diffuse to the plasma membrane through AQP3 [92].

### 3.4. Immune Function

Wound healing is a complex process. In addition to the aforementioned antioxidant, antibacterial, and anti-inflammatory properties, immunity also plays a very important role. A variety of important immune cells and immune molecules are involved, and the in-depth study of their mechanisms can guide clinical targeted therapy to promote wound repair. The immunomodulatory effect of propolis is mainly manifested in three aspects, namely, its effect on macrophages, lymphocyte-level antibody production, and antitumor activity [93]. In immune cells, antigen presentation, phagocytosis, cytokine production, and inflammation are closely related to macrophages, and they play an important role in the immune system. Some researchers used wax-free and fully water-soluble derivative (WSD) to conduct bacterial experiments first, and then to detect TNF activity. After using WSD, it can change the hemolysis in the serum. It can stimulate the macrophages in the abdominal cavity to produce other mediators, which is also consistent with the decrease in NBT and the increase in total protein secretion [94]. Studies have shown that the six compounds separated and identified from Brazilian propolis can improve the fluidity and dispersion of macrophages [95]. The effects of propolis extract and several other substances on human basic immune cells were studied, and the DNA synthesis and production of different types of cytokines by mitogen-activated peripheral blood mononuclear cells (PBMC) and purified T lymphocytes were tested impact. The results show that monocytes/macrophages (IL-1*β*, IL-12) and Th1-type (IL-2) and Th2-type (IL-4) lymphocytes produce cytokines which are inhibited, while T regulatory cells produce TGF-*β*1 in a rising state. The above experimental results prove that propolis has a direct regulatory effect on the basic functional characteristics of immune cells, which may be mediated by the Erk2 MAP kinase signaling pathway. Therefore, bee propolis can be regarded as a powerful natural inflammatory drug, which may affect different types of immune responses through immune regulatory T cells [96].

### 3.5. The Role of Mast Cells in Wound Healing

Mast cells are involved in three phases of wound healing: inflammatory phase, proliferative phase, and remodeling phase [97–99]. When the body is traumatized, one of the first cell types to respond is mast cells, which are a large number of inflammatory cells present in the body [100]. It mainly includes histamine, VEGF, interleukin IL -6, and IL-8, which help to increase endothelial permeability and vasodilation, and to promote the migration of monocytes and neutrophils to the wound site [101]. During inflammation, mast cells first aggregate to the wound injury site, where they mediate monocytes, followed by neutrophils, releasing all mediators. During the proliferative phase, mast cells interact with keratinocytes to elevate keratinocytes from the basement membrane and migrate into the wound. Then interact with fibroblasts, and fibroblasts will release some growth factors to promote wound healing. Finally, the effect on angiogenesis, mainly a regulatory effect, is that mast-cell-derived mediators contribute to neovascularization, fibrinogenogenesis or re-epithelialization during repair. In the remodeling phase, it is primarily the role played by other cells recruited by mast cells, such as macrophages, which play a role in re-epithelialization, fibroblast proliferation, and remodeling through the release of FGF and TGF-*β* [102]. Caffeic acid phenethyl ester (CAPE), the active ingredient in propolis, can reduce the release of histamine and the production of inflammatory factors in wound healing, as well as the release of locally induced vasoactive substances [103, 104]. Chrysin and kaempferol are previously reported flavonoid compounds that inhibit mast cell release of chemical mediators and cytokines, such as IL-4, IL-13 [105–107]. The ethanolic extract of Chinese propolis is the strongest inhibitor of mast cell degranulation, and chrysin and kaempferol are also the active ingredients in propolis ethanol extract. Chrysin also inhibits cytokine production by mast cells after antigenic stimulation [108] and reduces histamine release from mast cells [109]. Treatment of oral surgical wounds with propolis and dexamethasone to compare their effects on mast cells around the wound. Compared with dexamethasone, the number of mast cells in the wound treated with propolis was reduced, and the wound treatment showed a good anti-inflammatory effect [110]. Zinc and mast cells induce inflammatory cells (such as skin fibroblasts) to produce IL-6, which plays a key role in wound healing and promotes wound healing by activating gpr39/IL-6 signal axis [102].

## 4. Synergism between Propolis and Other Drugs

Many scholars have made propolis into different forms of wound dressings, such as foam, polyurethane, nano-propolis fibers, hydrogels, and so on. Antibacterial activity is one of the main physiological activities of propolis, and it plays an important role in promoting wound healing. The combination of propolis and antibiotics is used frequently. For example, Brazilian red propolis (BZP-BRP) and fluconazole are used to evaluate the ability to show resistance to *Candida glabrata* . In order to analyze the development of drug resistance, these fungal drug-sensitive strains were cultured in fluconazole and Brazilian red propolis (BZP-BRP). The laboratory results showed that *Candida* was resistant to various antifungal drugs. Brazilian red propolis (BZP-BRP) is not only active against resistant strains, but also does not induce resistance. In addition, the synergy between the two was studied by the chessboard method, and the results showed that for most isolates, Brazilian red propolis and fluconazole have a synergistic effect [88]. Propolis (collected from Brazil and Bulgaria) and antibiotics (chloramphenicol, tetracycline, and neomycin acting on ribosomes) may have a synergistic effect on *Salmonella typhi* in vitro. The synergy is studied by using the sum of the minimum inhibitory concentrations of propolis and these antimicrobial agents, and the number of living cells is evaluated according to the culture time. Brazilian propolis has antibacterial effect on *Salmonella typhi*, while Bulgarian propolis has bactericidal activity and has synergistic effects with three antibiotics [111].

The antibacterial properties of ethanol extracts of 13 propolis samples from different regions of Serbia on 39 microorganisms were studied, and the synergistic effect of propolis and antibacterial drugs was measured on agar containing sub-inhibitory concentration of propolis by the disc diffusion method. Propolis ethanol extract exhibits synergistic effects with selected antibiotics and shows the ability to enhance antifungal activity. This indicates that the antibacterial potential of propolis alone or in combination with certain antibiotics and antifungal drugs has potential medical value [112]. Experimental studies have shown that the ethanol extract of propolis with strong antibacterial activity has significant synergistic effect on the antibacterial activities of streptomycin and cloxacillin and has moderate synergistic effect on other antibacterial activities except ampicillin [113]. In addition, the combined use of propolis and drugs also has a certain therapeutic effect on cancer cells. Some researchers have focused on the effects of photodynamic therapy mediated by propolis and radachlorin on human head and neck cancer cells AMC-HN-4. After administration of propolis and radachlorin, laser irradiation was performed, and the viability of AMC-HN-4 cells was analyzed by MTT method. The final results show that compared with photodynamic therapy or propolis alone, the combined use of propolis can significantly enhance cell apoptosis and anti-proliferation effects [114].

The above experimental data and results all show that the combination of propolis and other compounds has a synergic effect on the treatment, and antibacterial activity of cancer cells, and better promotes the effect of the drug.

## 5. Conclusions

When people realize the benefits of propolis to human beings, scientists at home and abroad have done a lot of research on propolis. The chemical components of propolis are very complex, and different chemical components play different roles. At present, propolis has been widely used in food, health products, cosmetics, and beauty products and has a broad market and application value.

Propolis is rich in flavonoids, polyphenols, terpenoids, aromatic acids, and other pharmacological active ingredients. Flavonoids can promote the synthesis of collagen, and flavonoids and other ingredients also have antibacterial and anti-inflammatory functions. In skin wound healing, propolis can reduce scar formation, shorten healing time, increase wound contraction, accelerate tissue repair, and ultimately improve the quality of life of patients. It can be seen that the importance of propolis to the human body is extreme. In order for my country's propolis products to win more shares in the international market, it is necessary to conduct more in-depth discussions on some issues in the research, development and application of propolis. For example, first, there is little research on the combination of propolis and other substances. In this regard, it can be increased to use propolis with low toxicity with other drugs to play a greater medicinal value. Second, propolis can be made into different dosage forms for clinical use. At present, there is little research on intelligent materials and nano-materials using propolis, which will be a very important research direction in the future research. Third, propolis can be further purified and optimized, and the role of each effective substance can be brought into full play.

At present, some of the mechanism of propolis is not perfect, and there are many directions worthy of research and discussion. This article only reviews the effects and mechanisms of propolis on wound healing and the effects of propolis and other compounds in order to provide more effective and comprehensive information and provide some ideas for the development and utilization of propolis in the future.

## Figures and Tables

**Figure 1:** Chemical structural formula of some active ingredients in propolis.

**Figure 2:** The mechanism of propolis on wound healing. IL-6—interleukin-6, iNOS—inducible nitric oxide synthase, NO—nitric oxide, TGF-*β*—transforming growth factor-*β*, VEGF—vascular endothlial growth factor, Th1—helper T 1, Th2—helper T 2, SOD—superoxide dismutase, MDA—malondialdehyde.

**Table 1:** Treatment of other diseases with propolis.

S. No	Propolis type	Medical applications	Mian result	References
1	Green, red, or brown propolis	Atherosclerosis	Reduce atherosclerotic lesion area regulating inflammatory and angiogenic factors	[15]
2	Istanbul, Turkey propolis	Diabetes	Decrease of blood glucose significant improvement in pancreas, liver and kidney tissue	[16]
3	Brazilian extract of propolis (EEP)	Oral health	Effectively remove dental improve marginal periodontal tissue	[17]
4	Propolis	Radiation resistance	Inducing apoptosis increase the phosphorylation of Akt/mTOR and hinder cell migration	[18]
5	Brazilian propolis	Anti-ulcer effect	Inhibition of diclofenac induced ulcer formation antagonism to histaminergic system	[19]
6	Trigona sp. propolis	Dental pulp disease	Inhibition of IL-6 expression in dental pulp of inflammatory rats	[20]
7	Brown propolis from Southern Brazil	Anti-angiogenesis	Inhibition of tubular structure formation of endothelial cells on matrix gel (tubulogenesis)	[21]
8	Australian propolis extract (AP-1)	Antitumor activity	Promoting apoptosis and enhancing the anticancer activity of dox promote necrosis reversion to programmed cell death	[22]
9	Ethanol-soluble derivative of propolis	Protect liver activity	Elimination of hepatic collagen deposition, inflammatory signals and oxidative stress	[23]
10	Propolis extract	Vaginal use	Reorganization of vaginal mucosa faster organizational recovery decreased inflammatory response	[24]
11	Tekirdag-Turkey propolis	Antitumor activity	Activation of caspase cascade pathway induces apoptosis in C6 glioma cells	[25]
12	Ethanolic extract of propolis of Chihuahua (EEPCh)	Hypoglycemic effect	Significantly inhibited the increase of blood glucose and weight loss in diabetes mice	[26]
13	Populus-type propolis raw materials	Regulating blood lipids	Improvement of carotid restenosis in hypercholesterolemic rabbits inhibit neointimal hyperplasia reduce blood lipid level enhance antioxidant activity	[27]
14	Tehran, Iran propolis	Cardioprotective effect	Reduce oxidative stress, myocardial enzymes, histopathological degeneration and COX-2 expression in myocardial tissue	[28]
15	Korean propolis	Gastrointestinal diseases	Inhibit MAPK and NF-*κ*B signal activation effectively inhibited the pro-inflammatory response induced by *Helicobacter pylori*	[29]

**Table 2:** Effects of different forms of propolis on wound healing.

S. No	Propolis form	Experimental model	Main results	References
1	Propolis ointment	Square skin incision	Affect stimulating keratinocytes cell proliferation	[30]
2		Diabetic foot ulcer	Reduced ulcer area enhanced wound healing	[31]
3		Pulp wound	Maintain low inflammation and microbial cell population stimulating restorative dentin	[32]
4		Burn	Stimulates the accumulation of glycosaminoglycans on the wound surface required for granulation, tissue growth and wound closure to accelerate the repair of burn tissue	[33]
5		Chronic wound	Treatment of chronic wound infection caused by *Proteus mirabilis*	[34]
6		Cell CRL-7522	Enhance the proliferation, activation and growth of skin cells	[35]
7		Rat skin wound	Speed up wound healing high inflammatory cell infiltration rate higher granulation tissue	[36]

8	Propolis extract	Tooth pulp wound	Dentin tubules are arranged more orderly as pulp capping agent	[37]
9		Skin wound	*Staphylococcus aureus* and *Staphylococcus epidermidis* have inhibitory effects improve skin antibacterial effect	[38]
10		Damage caused by striking	Contains fibroblasts and collagen a large number of mitotic cells stimulate cell proliferation and tissue repair	[39]
11		Wound (about 11 mm)	Accelerate wound healing improve collagen deposition	[40]

12	Wound dressing containing propolis	Third degree burn wound	The area of the burn was reduced no inflammation and edema	[41]
13		Back incision	Fibroblast proliferation contributes to collagen deposition increased synthesis of natural hyaluronic acid	[42]

14	Propolis contains biocellulose membrane	Back and neck trauma	Wound healing improved fibroblast and collagen production increased	[43]
15		Wound (about 6 mm)	Tissue repair of contaminated wounds shorter time and better effect	[44]
16	Propolis and metal nanoparticles and biology medical thread combination	Surgically infected wound	Promote cell migration and proliferation gives effective antibacterial power to surgical sutures	[45]

**Table 3:** Study on anti-inflammatory mechanism of propolis promoting wound healing.

S. No	Propolis administration mode	Trauma model	Action effect	References
1	External application	Burn	Accelerate the tissue repair process reduced local inflammation	[49]

2	Drip	Alkali burns of rabbit cornea	Decreased infiltration of inflammatory cells	[67]

3	Apply	Six traumas in diabetic mice	Reduce neutrophil infiltration normal macrophages in wound tissue	[68]
4		Superficial second-degree burn	Reduced inflammation rapid wound healing	[69]
5		Skin wounds in diabetic mice	Increase in damage shrinkage reduction of inflammatory symptoms	[70]

**Table 4:** Study on antibacterial mechanism of propolis in promoting wound healing.

S. No	Propolis administration mode	Trauma model	Action effect	References
1	Apply	Oral cavity	Antibacterial activity against *Streptococcus mutans* reduced the proliferation of biofilms	[76]

2	External application	Trauma model	*Staphylococcus aureus* has inhibitory effect	[77]
3		Rat wound	The antibacterial activity of *Escherichia coli* and *Staphylococcus aureus* was enhanced	[78]

4	Drip		All three propolis had inhibitory effects on *Streptococcus albicans*	[79]

**Table 5:** Study on antioxidant mechanism of propolis in promoting wound healing.

S.NO	Propolis administration mode	Trauma model	Action effect	References
1	Oral	Gastric ulcer	Increased mucin production proliferation of mucosal cells reconstruction of oxidation balance	[84]
2		Esophageal burn in mice	Reduced lipid peroxidation promotes the recovery of antioxidant enzyme activity	[85]

3	Apply	Deep burns	Increase the content of SOD in serum	[86]
